The article "Silencing microRNA-27a inhibits proliferation and invasion of human osteosarcoma cells through the SFRP1-dependent Wnt/β-catenin signaling pathway" was retracted in 2026. Reasons: plagiarized data; plagiarized images; overlap with other authors' work; concerns about the data.

# Silencing microRNA-27a inhibits proliferation and invasion of human osteosarcoma cells through the SFRP1-dependent Wnt/β-catenin signaling pathway

**DOI:** 10.1042/BSR20182366

**Published:** 2019-06-04

**Authors:** Yu Mu, Lina Zhang, Xue Chen, Si Chen, Yuanyuan Shi, Junfeng Li

**Affiliations:** 1 Department of Colorectal Surgery, The Second Hospital of Jilin University, Changchun 130041, P.R. China; 2 Department of Orthopedics, The Second Hospital of Jilin University, Changchun 130041, P.R. China; 3 Department of Geriatrics, The Second Hospital of Jilin University, Changchun 130041, P.R. China; 4 Department of Nursing, The Second Hospital of Jilin University, Changchun 130041, P.R. China; 5 Department of Clinical Laboratory, The Second Hospital of Jilin University, Changchun 130041, P.R. China

**Keywords:** Invasion, MicroRNA-27a, Osteosarcoma, Proliferation, SFRP1, Wnt/β-catenin signaling pathway

## Abstract

Osteosarcoma is the most common malignant tumor of bone with a high potential for metastasis. Importantly, microRNA-27a (miR-27a) is involved in the progression of osteosarcoma. The present study aims to discuss the effects of miR-27a and its target gene secreted frizzled related protein 1 (*SFRP1*) on proliferation and invasion of human osteosarcoma cells via Wnt/β-catenin signaling pathway. The expression of miR-27a and SFRP1 in osteosarcoma tissues and cells was detected, followed by identification of their relations. Subsequently, miR-27a mimic, miR-27a inhibitor, or siRNA against SFRP1 were introduced into cells (HOS and U2OS) to investigate their role in cell proliferation and invasion. The expression of Wnt/β-catenin signaling pathway-related gene was analyzed to further uncover the regulatory mechanism of miR-27a. The osteosarcoma tissues and cells exhibited elevated miR-27 expression and reduced SFRP1 expression. SFRP1 was verified to be a target gene of miR-27a. Meanwhile, silenced miR-27a inhibited proliferation and invasion of human osteosarcoma cells. Finally, silencing miR-27a inhibited the activation of Wnt/β-catenin signaling pathway, evidenced by reduced β-catenin expression. Our study draws a conclusion that silencing miR-27a dampens osteosarcoma progression, which might be achieved through the inactivation of the Wnt/β-catenin signaling pathway by up-regulating SFRP1.

## Introduction

Osteosarcoma, one of the most common primary bone tumors, is a sort of invasive tumor which mainly affects adolescents [1]. Annual morbidity rate of osteosarcoma is approximately 0.3–0.5 per 10 million people across the world, and it presents a bimodal age distribution with peaks at 15–19 and 70 years [2,3]. Osteosarcoma is typically characterized by local pain, weight loss, fever, facial paleness, asitia and dysfunction [4,5]. At present, it is acknowledged that this disease is mainly caused by genetic factors and environmental factors [3,6]. Conventional therapies for patients who were diagnosed with osteosarcoma include surgical resection, chemotherapy, radiotherapy and immunotherapy [7]. However, resistance to these therapies often results in poor prognosis of patients with osteosarcoma, moreover, drug-resistant phenotypes in frequent acquisition manner and ‘secondary malignancies’ occurrence are crucial barriers to obtain satisfying consequences [8]. It is reported that some microRNAs (miRNAs) crucially affect the occurrence and development of tumors [9]. MiRNAs refer to non-coding small molecular RNAs with a length of 18–23 nucleotides, and it is confirmed to be involved in a series of biological processes, and some specific miRNAs have been found that may affect metastasis of osteosarcoma [10]. Therefore, it is of great interest to explore more roles of specific miRNAs in osteosarcoma.

The article "Silencing microRNA-27a inhibits proliferation and invasion of human osteosarcoma cells through the SFRP1-dependent Wnt/β-catenin signaling pathway" was retracted in 2026. Reasons: plagiarized data; plagiarized images; overlap with other authors' work; concerns about the data.

MicroRNA-27a (miR-27a), a member of the miR-23a-27a-24-2 cluster, is identified as the miRNA of a sort of cancer gene [11]. As a major member among the miRNAs family, miR-27a not only is involved in the regulation of osteoblast proliferation, apoptosis and differentiation, bone formation, but also plays an oncogenic role in different types of tumors [12,13]. Moreover, recent researches have revealed that miR-27a plays an essential part in promoting the proliferation, migration and invasion of human osteosarcoma cells, and therefore advances the rapid progression of osteosarcoma [13,14]. Previously, another up-regulated miRNA, miR-940, was suggested to enhance human osteosarcoma cell abilities of proliferation, migration and invasion while suppressing apoptosis via secreted frizzled related protein 1 (SFRP1) down-regulation through Wnt/β-catenin signaling pathway activation [15]. SFRP1 belongs to the SFRP family with a region homologous to the recognized Wnt-binding site of frizzled proteins, and its gene *SFRP1* has been identified as a tumor suppressor gene [16]. SFRP1 can block the Wnt signaling pathway by interrupting the interaction between Wnt glycoprotein (ligand) and frizzled receptor, thus being a negative regulatory factor of the Wnt signaling pathway [17]. In recent years, abnormal activation of the Wnt signaling pathway is reported to be related to tumor formation; as a negative regulator in the Wnt signaling transduction, SFRP1 may play a significant role in tumor occurrence [18]. Wang et al. [19] found that miR-27a might target SFRP1 to regulate the Wnt/β-catenin signaling pathway in glioma. Additionally, it has previously reported the mechanism that miR-27a regulated the progression of colon cancer by targeting SFRP1 via the Wnt/β-catenin signaling pathway [20]. This paper proposes a hypothesis that miR-27a might have an effect on osteosarcoma in relation to SFRP1 and the Wnt/β-catenin signaling pathway. For this reason, this study detected effect of miR-27a on osteosarcoma through regulating the Wnt/β-catenin signaling pathway by targeting SFRP1.

The article "Silencing microRNA-27a inhibits proliferation and invasion of human osteosarcoma cells through the SFRP1-dependent Wnt/β-catenin signaling pathway" was retracted in 2026. Reasons: plagiarized data; plagiarized images; overlap with other authors' work; concerns about the data.

## Materials and methods

### Study subjects

The present study included 102 patients (67 males and 35 females with a mean age of 20 years, ranging from 10 to 51 years) pathologically diagnosed with primary osteosarcoma and underwent surgical resection in the Second Hospital of Jilin University between October 2013 and September 2015. Among all the patients, 40 patients had the age of <20 years, and 62 patients had the age of ≥20 years. For tumor size, there were 43 patients with tumors less than 8 cm and 59 patients with tumors greater than 8 cm. As for tumor location, 63 patients were observed with tumors located in the femur and 39 patients with tumors located in the tibia. There were 54 patients with highly and moderately differentiated tumors and 48 patients with poorly differentiated tumors. Based on Enneking staging [21], there were 54 patients with Enneking stage I osteosarcoma, and 48 patients with Enneking stage II osteosarcoma. Osteosarcoma and adjacent normal fibrous connective tissues were obtained from all patients immediately after surgical resection of osteosarcoma, and were stored in Eppendorf (EP) freezing tubes. Pathological and histological analysis after surgery was performed for all tissue specimens, and all patients were diagnosed as primary osteosarcoma with osteoblasts as the main type.

### Successful construction of plasmids

Polymerase chain reaction (PCR) amplification was applied for sequences within 3′-untranslated region (3′-UTR) of human SFRP1. After PCR amplification, sequences within 3′-UTR of SFRP1 were inserted into the pGL3 plasmid (Promega Corp., Madison, Wisconsin, U.S.A.) by digestion with XbaI restriction enzyme to obtain pGL3-WT-SFRP1-3′-UTR (WT-SFRP1) plasmid. Meanwhile, pGL3-MUT-SFRP1-3′-UTR (MUT-SFRP1) plasmid was constructed with sequences (containing the mutant locus of miR-27a-binding site within the 3′-UTR of SFRP1). PCR primer sequences of SFRP1-3′-UTR were as follows: 5′-end-sequence, 5′-AAAGCAAGGGCCATTTAGATTAG; 3′-end-sequence, 5′-TTCTGGGCTTGACCTTAATTGTA. Enzyme digestion was performed at 37°C for 6 h. The miR-27a mimic (5′-UUCACAGUGGCUAAGUUCCGC-3′), control mimic (5′-UUGUACUACACAAAAGUACUG-3′), miR-27a inhibitor (5′-GCGGAACUUAGCCCACUGUGAA-3′) and control inhibitor (5′-CAGUACUUUUGUGUAGUACAA-3′) were purchased from Shanghai GenePharma Co., Ltd. (Shanghai, China). The SFRP1 siRNA (si-SFRP1) and negative control siRNA (si-NC) were bought from Invitrogen Inc. (Carlsbad, CA, U.S.A.).

The article "Silencing microRNA-27a inhibits proliferation and invasion of human osteosarcoma cells through the SFRP1-dependent Wnt/β-catenin signaling pathway" was retracted in 2026. Reasons: plagiarized data; plagiarized images; overlap with other authors' work; concerns about the data.

### Cell treatment

Human osteosarcoma cell lines (HOS and U2OS) and normal osteoblast cell line (hFOB1.19) from the cell bank of the Chinese Academy of Sciences (Shanghai, China) were cultured in 90% Dulbecco’s modified Eagle’s medium (DMEM) (Gibco, Grand Island, NY, U.S.A.) containing 10% fetal bovine serum (FBS) (Gibco, Grand Island, NY, U.S.A.). Upon reaching 90% confluence, cells were transfected in accordance with the instructions of Lipofectamine 2000 kit (LF2000; Invitrogen, Carlsbad, CA, U.S.A.). Osteosarcoma cells (HOS, U2OS) were transfected with miR-27a inhibitor, miR-27a mimic, SFRP1 siRNA plasmids, or pathway inhibitor Dickkopf-1 as well as the corresponding controls.

### RNA isolation and quantitation

Total RNA was extracted with the RNAiso Plus kit (Takara, Biotechnology Ltd., Dalian, China). Reverse transcription was performed with the PrimeScript RT reagent kit (Takara, Biotechnology Ltd., Dalian, China). The reverse transcription quantitative PCR (RT-qPCR) was conducted using SteponePlus (ABI Company, Oyster Bay, NY) PCR instrument [19]. The relative expression of SFRP1 (Gene ID: 6422) and miR-27a was examined, with *β-actin* (Gene ID: 2597) used as an internal reference. The primer sequences are shown in Table 1.

**Table 1:** Primer sequences for RT-qPCR

	5′ end	3′ end
SFPR1	CGAGTTTGCACTGAGGATGA	CAGCAAGCTTCTTCAGGTC
miR-27a	TTCACAGTGGCTAAG	GTGCAGGGTCCGAGGT
β-actin	TGGCACCCAGCACAATGAA	CTAAGTCATAGTCCGCCTAGAAGCA

### Western blot analysis

Total protein was extracted. With the addition of 10% SDS/PAGE, 20 μg protein samples were added into each well. Next, samples were added with primary antibody rabbit polyclonal anti-SFRP1, vascular endothelial growth factor (VEGF), c-Myc, cyclin D1 and β-catenin (Santa Cruz Biotechnology Inc., Santa Cruz, CA, U.S.A.), and incubated at 4°C overnight. The next day, samples were incubated with secondary antibody POD–conjugated goat anti-rabbit antibody (1:5000) at room temperature for 30 min and then added with horseradish peroxidase (HRP, Bio-Rad Laboratories, Hercules, CA, U.S.A.) for developing. The intensity of protein bands was analyzed by Image Quant 350 and Image Quant TL-1 (GE Healthcare, Fairfield, CT, U.S.A.), with β-actin as the internal reference.

### Dual-luciferase reporter gene assay

The analysis for potential target genes of miR-27a was performed with online biological software, including TargetScan (http://www.targetscan.org/), PicTar (http://pictar.mdc-berlin.de/) and microRNA.org (http://www.microrna.org/). The clonal expansion was performed for sequences containing miR-27a-binding site within the 3′-UTR of SFRP1. The PCR products were cloned into the downstream of luciferase gene in the pmirGLO plasmid (Promega Corp., Madison, Wisconsin, U.S.A.). With a mutation of miR-27a-binding site of *SFRP*1, the pRL-TK plasmid (*Renilla* luciferase-thymidine kinase; TaKaRa, Holdings Inc., Kyoto, Japan) that expressed *Renilla* luciferase activity (Rel value) was selected as an internal reference to adjust the number of cells and transfection efficiency. After cell transfection using Lipofectamine RNAiMAX Kit (Thermo Fisher Scientific Inc., Waltham, MA, U.S.A.), osteosarcoma cells (HOS, U2OS) were co-transfected with WT-SFRP1 and miR-27a inhibitor plasmids, MUT-SFRP1 and miR-27a inhibitor plasmids, WT-SFRP1 and control inhibitor plasmids or MUT-SFRP1 and control inhibitor plasmids. Forty-eight hours later, the activity of luciferase was analyzed by Dual-Luciferase Reporter Assay System (Promega, Corp., Madison, Wisconsin, U.S.A.).

The article "Silencing microRNA-27a inhibits proliferation and invasion of human osteosarcoma cells through the SFRP1-dependent Wnt/β-catenin signaling pathway" was retracted in 2026. Reasons: plagiarized data; plagiarized images; overlap with other authors' work; concerns about the data.

### 3-(4,5-dimethylthiazol-2-yl)-2,5-diphenyltetrazolium bromide assay

HOS and U2OS cells were cultured in a 96-well plate (1 × 10^5^ cells/well). These cells were separately transfected with miR-27a inhibitor plasmid and control inhibitor plasmid (Shanghai GenePharma Co., Ltd., Shanghai, China), with four replicates set in each group. After 24, 48, 72, and 96 h of cell transfection, Vybrant® MTT Cell Proliferation Assay Kit (Thermo, U.S.A.) was applied to detect cell proliferation [22].

### Transwell assay

A total of 600 μl medium containing tumor cells (HOS and U2OS) were added into the basolateral chamber of the Matrigel-coated Transwell chambers (Corning Costar, Tewksbury, MA, U.S.A.), and serum-free medium containing 5 × 10^4^ tumor cells was added into the apical chamber. After 24-h culture at 37°C, with serum-free medium sucked away, cells attached to the upper surface of chamber were removed. The rest of cells was fixed with 100% methyl alcohol, and then stained with Crystal Violet. The number of cells invading Matrigel was counted in three random fields.

### Immunofluorescence staining

Cells cultured on cover glass coated with 0.1% gelatin in a six-well plate were fixed with 4% paraformaldehyde for 20 min, and then sealed with phosphate buffer saline-Tween 20 (PBST) containing 10% goat serum at room temperature for 1 h. Added with primary antibody rabbit polyclonal anti-β-catenin (Abcam, Cambridge, MA, U.S.A.), cells were incubated at room temperature for 30 min, and then incubated at 4°C overnight. After being washed by PBST three times, cells were added with secondary antibody fluorescein isothiocyanate (FITC)-conjugated goat anti-rabbit (1:5000) and added with 4′,6-diamidino-2-phenylindole (DAPI) to label cell nucleus. Next, the cover glass was inverted on a glass slide, followed by observation under a confocal microscope.

The article "Silencing microRNA-27a inhibits proliferation and invasion of human osteosarcoma cells through the SFRP1-dependent Wnt/β-catenin signaling pathway" was retracted in 2026. Reasons: plagiarized data; plagiarized images; overlap with other authors' work; concerns about the data.

### TOP-FLASH reporter assay

TOP-FLASH reporter assay was applied to detect the activity of the Wnt-β-catenin signaling pathway, in which β-catenin enters into the nucleus to form a complex with the transcription factor T-cell factor (TCF)/lymphoid enhancer-binding (LEF) regulating the transcription of downstream gene expression. Cell densities of HOS cells and U2OS cells were separately adjusted to 1 × 10^5^ cells/ml using DMEM. Then these cells (500 μl per well) were inoculated into a 24-well plate, followed by transfection based on the instructions of the Lipofectamine 2000 kit (LF2000; Invitrogen, Carlsbad, CA, U.S.A.) when cells reached 80–90% confluence. Cells transfected with miR-27a inhibitor, miR-27a mimic, SFRP1 siRNA plasmids as well as their corresponding controls were separately co-transfected with TOP-flash plasmid and pRL-TK plasmid. After 48 h of transfection, cells were added with 200 μl prepared passive lysis buffer (PLB, 1:4) and centrifuged for 3 min (12000 rpm, 4°C). Then supernatant (10 μl) was obtained, followed by centrifugation for 1 min (12000 rpm, 4°C). The luciferase assay reagent II (LAR II) and Stop & Glo reagent were used to detect Luc (Firefly luciferase activity) and Rel values. The transcriptional activity of TCF/LEF was visualized by the ratio of TOP-Flash Luc/Rel value (Ratio of TOP-Luc/Rel).

### Statistical analysis

Statistical analysis was performed by SPSS 20.0 software (IBM Corp. Armonk, NY, U.S.A.). Measurement data were presented as mean ± standard deviation (S.D.). Comparisons of data between two groups were analyzed by independent sample *t* test, and among multiple groups were analyzed by one-way analysis of variance (ANOVA). Repeated-measures ANOVA was used in the comparison of data at different time points. *P*<0.05 was considered statistically significant.

## Results

### Highly expressed miR-27a and lowly expressed SFRP1 in osteosarcoma tissues and cells

According to the results of RT-qPCR and Western blot analysis, miR-27a expression in osteosarcoma tissues was increased and mRNA and protein expression of SFRP1 was declined compared with those in the adjacent normal fibrous connective tissues (all *P*<0.05) (Figure 1). Compared with the normal osteoblast cell line (hFOB1.19), osteosarcoma cell lines (HOS and U2OS) also exhibited higher miR-27a expression and lower mRNA and protein expression of SFRP1 (all *P*<0.05) (Figure 2). These results suggested that increased miR-27a expression and decreased SFRP1 could be associated with osteosarcoma progression.

The article "Silencing microRNA-27a inhibits proliferation and invasion of human osteosarcoma cells through the SFRP1-dependent Wnt/β-catenin signaling pathway" was retracted in 2026. Reasons: plagiarized data; plagiarized images; overlap with other authors' work; concerns about the data.

**Figure 1:** Increased miR-27a expression and decreased SFRP1 in osteosarcoma tissues (**A**) miR-27a expression in osteosarcoma and adjacent normal fibrous connective tissues by RT-qPCR. (**B**) mRNA expression of SFRP1 in osteosarcoma and adjacent normal fibrous connective tissues by RT-qPCR. (**C**) Protein bands of SFRP1 and GAPDH in osteosarcoma and adjacent normal fibrous connective tissues by Western blot analysis. (**D**) Protein expression of SFRP1 in osteosarcoma and adjacent normal fibrous connective tissues by Western blot analysis. There were 102 samples in the experiment. The measurement data were expressed as mean ± S.D. The comparison between two groups was analyzed by *t* test. *P<0.05 compared with the adjacent normal fibrous connective tissues. Abbreviation: GAPDH, glyceraldehyde-3-phosphate dehydrogenase.

**Figure 2:** Increased miR-27a expression and decreased SFRP1 in osteosarcoma cell lines (HOS and U2OS) (**A**) miR-27a expression in osteosarcoma (HOS and U2OS) and normal osteoblast (hFOB1.19) cells by RT-qPCR. (**B**) *SFRP1* mRNA expression of SFRP1 in osteosarcoma (HOS and U2OS) and normal osteoblast (hFOB1.19) cells by RT-qPCR. (**C**) Protein bands of SFRP1 and GAPDH in osteosarcoma (HOS and U2OS) and normal osteoblast (hFOB1.19) cells by Western blot analysis. (**D**) Protein expression of SFRP1 in osteosarcoma (HOS and U2OS) and normal osteoblast (hFOB1.19) cells. The measurement data were expressed as mean ± S.D. The comparison among multiple groups was analyzed by one-way ANOVA; the experiment was repeated three times. *P<0.05 compared with the normal osteoblast (hFOB1.19) cells. Abbreviation: GAPDH, glyceraldehyde-3-phosphate dehydrogenase.

### miR-27a and SFRP1 expression is related to the degree of tumor differentiation and Enneking staging of patients with osteosarcoma

Through analyzing the relationship between the expression of miR-27a and SFRP1 and the clinicopathological features of patients with osteosarcoma, it was found that miR-27a expression and mRNA and protein expression of SFRP1 were not associated with age, sex, tumor size and tumor location of osteosarcoma patients (all *P*>0.05), but were associated with the degree of tumor differentiation, and Enneking staging (both *P*<0.05) (Table 2).

**Table 2:** Associations of miR-27a expression and mRNA and protein expression of SFRP1 with clinicopathologic features of osteosarcoma patients

Clinicopathological features	*n*	miR-27a	*SFRP1* mRNA	SFRP1 protein
Age				
<20	40	1.89 ± 0.36	0.49 ± 0.11	0.67 ± 0.09
≥20	62	2.00 ± 0.42	0.46 ± 0.11	0.64 ± 0.10
Sex				
Male	67	1.93 ± 0.41	0.48 ± 0.13	0.66 ± 0.11
Female	35	2.02 ± 0.38	0.45 ± 0.12	0.64 ± 0.09
Tumor size (cm)				
<8	43	1.99 ± 0.46	0.46 ± 0.15	0.64 ± 0.11
≥8	59	1.94 ± 0.35	0.48 ± 0.11	0.66 ± 0.09
Tumor differentiation				
Well/moderate	54	1.71 ± 0.24^1^	0.55 ± 0.08^1^	0.72 ± 0.07^1^
Poor	48	2.24 ± 0.35^2^	0.38 ± 0.11^2^	0.57 ± 0.06^2^
Tumor location				
Femur	63	1.92 ± 0.36	0.48 ± 0.12	0.66 ± 0.10
Tibia	39	2.02 ± 0.45	0.45 ± 0.15	0.63 ± 0.10
Enneking stage				
Stage I	54	1.71 ± 0.24^1^	0.55 ± 0.08^1^	0.72 ± 0.07^1^
Stage II	48	2.24 ± 0.35^2^	0.38 ± 0.11^2^	0.57 ± 0.06^2^

There were 102 samples in the experiment. The measurement data were expressed as mean ± S.D. Comparison between the two groups was analyzed by *t* test, and among multiple groups was analyzed by one-way ANOVA. Different superscript numbers (1 and 2) indicated *P*<0.05.

The article "Silencing microRNA-27a inhibits proliferation and invasion of human osteosarcoma cells through the SFRP1-dependent Wnt/β-catenin signaling pathway" was retracted in 2026. Reasons: plagiarized data; plagiarized images; overlap with other authors' work; concerns about the data.

### miR-27a inhibits SFRP1 expression in HOS and U2OS cells

RT-qPCR and Western blot analysis were conducted to examine the expression of miR-27a and SFRP1 in HOS and U2OS cells. It showed that miR-27a expression was significantly decreased, but mRNA and protein expression of SFRP1 was elevated in cells transfected with miR-27a inhibitor in contrast with cells transfected with control inhibitor, while miR-27a expression was elevated but mRNA and protein expression of SFRP1 was decreased in the cells transfected with miR-27a mimic compared with cells transfected with control mimic (all *P*<0.05). Cells transfected with both miR-27a inhibitor and si-SFRP1 exhibited no significant difference in miR-27a expression but down-regulated mRNA and protein expression of SFRP1 in contrast with cells transfected with both miR-27a inhibitor and si-NC (*P*>0.05). But no significant difference was observed in miR-27a expression and mRNA and protein expression of SFRP1 among the cells without transfection, cells transfected with control inhibitor and control mimic (all *P*>0.05) (Figure 3). Therefore, it could be concluded that the expression of SFRP1 was suppressed by miR-27a.

**Figure 3:** The SFRP1 expression is inhibited by miR-27a in HOS and U2OS cells (**A**) miR-27a expression in HOS cells among seven groups detected by RT-qPCR. (**B**) miR-27a expression in U2OS cells among seven groups measured by RT-qPCR. (**C**) mRNA expression of SFRP1 in HOS cells among seven groups evaluated by RT-qPCR. (**D**) mRNA expression of SFRP1 in U2OS cells among seven groups determined by RT-qPCR. (**E**) Protein bands of SFRP1 and GAPDH in HOS cells among seven groups examined by Western blot analysis. (**F**) Protein bands of SFRP1 and GAPDH in U2OS cells among seven groups measured by Western blot analysis. (**G**) Protein expression of SFRP1 in HOS cells among seven groups examined by Western blot analysis. (**H**) Protein expression of SFRP1 in in U2OS cells among seven groups examined by Western blot analysis. The measurement data were expressed as mean ± S.D. The comparison among multiple groups was analyzed by one-way ANOVA; the experiment was repeated three times. *P<0.05 compared with the control inhibitor group; ^#^*P*<0.05 compared with the control mimic group; ^&^*P*<0.05 compared with the miR-27a inhibitor + si-NC group. Abbreviation: GAPDH, glyceraldehyde-3-phosphate dehydrogenase.

The article "Silencing microRNA-27a inhibits proliferation and invasion of human osteosarcoma cells through the SFRP1-dependent Wnt/β-catenin signaling pathway" was retracted in 2026. Reasons: plagiarized data; plagiarized images; overlap with other authors' work; concerns about the data.

### MiR-27a silencing inhibits the proliferation and invasion of HOS and U2OS cells by enhancing SFRP1

MTT (3-(4,5-dimethylthiazol-2-yl)-2,5-diphenyltetrazolium bromide) assay was conducted to examine the effect of miR-27a on proliferation of HOS and U2OS cells. After 24 h of transfection, cell viabilities of HOS and U2OS cells were examined every 24 h. After 24, 48, 72 and 96 h of cell transfection, cell proliferation in the cells transfected with miR-27a inhibitor was decreased compared with the cells transfected with inhibitor control, but was enhanced in cells transfected with miR-27a mimic in contrast with cells transfected with mimic control (all *P*<0.05). Besides, cells transfected with si-SFRP1 exhibited increased cell proliferation compared with cells transfected with si-control, and the similar trend was found in cells transfected with both miR-27a inhibitor and si-SFRP1 in contrast with cells transfected with both miR-27a inhibitor and si-NC (all *P*<0.05). Cell proliferation was similar among the cells without transfection, cells transfected with control inhibitor and control mimic (all *P*>0.05) (Figure 4A,B). These results showed that silenced miR-27a could reduce the proliferation ability of HOS and U2OS cells through up-regulating SFRP1.

**Figure 4:** Inhibited miR-27a suppresses the proliferation ability and invasion ability of HOS and U2OS cells through up-regulating SFRP1 (**A,B**) HOS and U2OS cell proliferation among seven groups after 24, 48, 72 and 96 h transfection examined by MTT assay. (**C**) HOS and U2OS cell invasion among seven groups detected by Transwell assay (×200). The measurement data were expressed as mean ± S.D. The comparison among multiple groups was analyzed by one-way ANOVA; the experiment was repeated three times. *P<0.05 compared with the control inhibitor group; ^#^*P*<0.05 compared with the control mimic group; ^@^*P*<0.05 compared with the si-control group; ^&^*P*<0.05 compared with the miR-27a inhibitor + si-NC group.

Transwell assay was performed to further evaluate the biological implications of miR-27a in invasion ability of HOS and U2OS cells after plasmid delivery. After 24 h of cell transfection, miR-27a inhibitor delivery induced a decreased invasion ability of HOS and U2OS cells in contrast with cells with control inhibitor transduction (all *P*<0.05). On the contrary, HOS and U2OS cells delivered with miR-27a mimic showed enhanced cell invasion in comparison with cells transduced with control mimic (*P*<0.05). Similarly, cells transduced with si-SFRP1 exhibited promoted cell invasion than cells transduced with si-control, and cells delivered with both miR-27a inhibitor and si-SFRP1 showed enhanced cell invasion than cells delivered with both miR-27a inhibitor and si-NC (all *P*<0.05). As for the cells without transfection, cells transfected with control inhibitor and control mimic, no significant difference in cell invasion was observed (all *P*>0.05) (Figure 4C). These results showed that silenced miR-27a could suppress the invasion ability of HOS and U2OS cells through up-regulating SFRP1.

The article "Silencing microRNA-27a inhibits proliferation and invasion of human osteosarcoma cells through the SFRP1-dependent Wnt/β-catenin signaling pathway" was retracted in 2026. Reasons: plagiarized data; plagiarized images; overlap with other authors' work; concerns about the data.

### SFRP1 is a target gene of miR-27a

Bioinformatics prediction regarding the potential relationship between miR-27a and SFRP1 suggested that miR-27a was of great potential to regulate SFRP1. Therefore, subsequent dual-luciferase reporter gene assay was performed to verify their relationship. After cell transfection, the luciferase activity of the HOS and U2OS cells transfected with both WT-SFRP1 and control inhibitor was set as 1. The cells transfected with both MUT-SFRP1 and miR-27a inhibitor and cells transfected with both MUT-SFRP1 and control inhibitor presented with no marked difference of luciferase activity, while cells with both WT-SFRP1 and miR-27a inhibitor transfection led to an evident increase in luciferase activity (*P*<0.05) (Figure 5). These results demonstrated that miR-27a could target SFRP1 by inhibiting its transcription.

**Figure 5:** miR-27a targets SFRP1 by inhibiting its transcription (**A**) The binding site of miR-27a and SFRP1 predicted by microRNA software. (**B**) Comparison of luciferase activity in HOS and U2OS cells after treatment with the WT-SFRP1 + miR-27a inhibitor, the MUT-SFRP1 + miR-27a inhibitor, the WT-SFRP1 + control inhibitor and the MUT-SFRP1 + control. WT-SFRP1, SFRP1 wild-type plasmid; MUT-SFRP1, SFRP1 mutant-type; *P<0.05 compared with the MUT-SFRP1 + miR-27a inhibitor, the WT-SFRP1 + control inhibitor and the MUT-SFRP1 + control groups. The measurement data were expressed as mean ± S.D. The comparison among multiple groups was analyzed by one-way ANOVA; the experiment was repeated three times.

### Silenced miR-27a inactivates the Wnt/β-catenin signaling pathway in HOS and U2OS cells by up-regulating SFRP1

The target relationship between miR-27a and SFRP1 was confirmed, but the specific molecular mechanism of miR-27a targeting SFRP1 in osteosarcoma through the Wnt/β-catenin signaling pathway was unclear. Therefore, mimic, inhibitor or siRNA against SFRP1 was delivered into HOS and U2OS cell to interfere with the expression of both miR-27a and SFRP1, with their effects analyzed through the detection on β-catenin mRNA and protein expression. The images revealed that β-catenin was not translocated into the nucleus of HOS and U2OS cells without transfection as well as cells delivered with control inhibitor and control mimic. However, β-catenin expression was increased in HOS and U2OS cells after miR-27a mimic transfection in comparison with cells transfected with control mimic, and β-catenin was translocated into the cell nucleus. Meanwhile, β-catenin expression in cells transfected with miR-27a inhibitor was significantly decreased than the cells transfected with control inhibitor (*P*<0.05). In contrast with the cells with both miR-27a inhibitor and si-SFRP1 transfection, cells transfected with both miR-27a inhibitor and si-NC showed increased β-catenin expression and β-catenin was translocated into the cell nucleus (*P*>0.05) (Figure 6A). Based on these results, we concluded that silenced miR-27a inactivated the Wnt/β-catenin signaling pathway in HOS and U2OS cells.

The article "Silencing microRNA-27a inhibits proliferation and invasion of human osteosarcoma cells through the SFRP1-dependent Wnt/β-catenin signaling pathway" was retracted in 2026. Reasons: plagiarized data; plagiarized images; overlap with other authors' work; concerns about the data.

**Figure 6:** miR-27a silencing inactivates the Wnt/β-catenin signaling pathway by up-regulating SFRP1 (**A**) Activities of the Wnt/β-catenin signaling pathway in HOS and U2OS cells detected by immunofluorescence staining (×400). (**B**) Ratio of TOP-Flash Luc/Rel in both HOS and U2OS cells among seven groups detected by TOP-FLASH reporter assay. (**C**) The protein bands of VEGF, c-Myc, cyclin D1 and GAPDH in HOS and U2OS cells among seven groups detected by Western blot analysis. The measurement data were expressed as mean ± S.D. The comparison among multiple groups was analyzed by one-way ANOVA; the experiment was repeated three times; *P<0.05 compared with the control inhibitor group; ^#^*P*<0.05 compared with the control mimic group; ^&^*P*<0.05 compared with the miR-27a inhibitor + si-NC group. Abbreviation: GAPDH, glyceraldehyde-3-phosphate dehydrogenase.

As shown in Figure 6B, no significant difference was observed in the ratio of TOP-Luc/Rel among HOS and U2OS cells without transfection as well as cells transfected with control mimic, control inhibitor and both si-SFPR1 and miR-27a inhibitor. The ratio of TOP-Luc/Rel was elevated in the cells delivered with miR-27a mimic in contrast with cells with control mimic transfection (*P*<0.05). The cells transfected with miR-27a inhibitor displayed significantly decreased ratio of TOP-Luc/Rel compared with cells transfected with control inhibitor, but cells delivered with both miR-27a inhibitor and si-SFPR1 exhibited increased ratio of TOP-Luc/Rel in contrast with cells transfected with both miR-27a inhibitor and si-NC (all *P*<0.05). Thus, these results suggested that silenced miR-27a might inactivate the Wnt/β-catenin signaling pathway by up-regulating SFRP1.

The article "Silencing microRNA-27a inhibits proliferation and invasion of human osteosarcoma cells through the SFRP1-dependent Wnt/β-catenin signaling pathway" was retracted in 2026. Reasons: plagiarized data; plagiarized images; overlap with other authors' work; concerns about the data.

Further, the results (Figure 6C) revealed that no obvious change in protein expression of VEGF, c-Myc and cyclin D1 was found among cells without transfection as well as cells transfected with control mimic and control inhibitor. The protein expression of VEGF, c-Myc and cyclin D1 was significantly higher in cells transfected with miR-27a mimic than cells with control mimic transfection, while was significantly lower in cells with miR-27a inhibitor transduction in contrast with cells transduced with control inhibitor (all *P*<0.05). Additionally, the protein expression of VEGF, c-Myc and cyclin D1 was significantly increased in cells delivered with both miR-27a inhibitor and si-SFPR1 compared with cells delivered with both miR-27a inhibitor and si-NC (all *P*<0.05). The results above led to a conclusion that silenced miR-27a inhibited the protein expression of VEGF, c-Myc and cyclin D1 in HOS and U2OS cells.

### Inactivated Wnt/β-catenin signaling pathway suppresses proliferation and invasion of HOS and U2OS cells

At last, to verify the effect of Wnt/β-catenin signaling pathway on the progression of osteosarcoma cells, comparison was conducted between cells transfected with miR-27a mimic and cells transfected with both miR-27a mimic and Dickkopf-1. It revealed that decreased cell proliferation, cell invasion and protein expression of VEGF, c-Myc and cyclin D1 in HOS and U2OS cells were found after both miR-27a mimic and Dickkopf-1 transduction compared with cells transduced with miR-27a mimic (*P*<0.05) (Figure 7). These findings suggested that cell proliferation and invasion could be suppressed by inhibiting Wnt/β-catenin signaling pathway.

**Figure 7:** Inactivation of Wnt/β-catenin signaling pathway inhibits proliferation and invasion of HOS and U2OS cells (**A**) Proliferation of HOS and U2OS cells after transfection with miR-27a mimic and with both miR-27a mimic and Dickkopf-1 examined by MTT assay. (**B**) Invasion of HOS and U2OS cells after transfection with miR-27a mimic and with both miR-27a mimic and Dickkopf-1 examined by Transwell assay (×200). (**C**) The protein bands of VEGF, c-Myc, cyclin D1 and GAPDH in HOS and U2OS cells after transfection with miR-27a mimic and with both miR-27a mimic and Dickkopf-1 examined by Western blot analysis. The measurement data were expressed as mean ± S.D. The comparison between two groups was analyzed by *t* test; the experiment was repeated three times; *P<0.05 compared with the miR-27a mimic group. Abbreviation: GAPDH, glyceraldehyde-3-phosphate dehydrogenase.

The article "Silencing microRNA-27a inhibits proliferation and invasion of human osteosarcoma cells through the SFRP1-dependent Wnt/β-catenin signaling pathway" was retracted in 2026. Reasons: plagiarized data; plagiarized images; overlap with other authors' work; concerns about the data.

## Discussion

The present study analyzed the effect of miR-27a on the proliferation and invasion of osteosarcoma cells. The luciferase assay verified that SFRP1 was the target gene of miR-27a. And miR-27a might activate the Wnt/β-catenin signaling pathway through targeting SFRP1, thereby to promote the proliferation and invasion ability of human osteosarcoma cells.

In the present study, miR-27a expression was increased in osteosarcoma tissues and cells, while that of SFRP1 were declined. Jones et al. [23] confirmed that miR-27a was highly expressed in osteosarcoma cells (HOS, KHOS, and U2OS) and the predicted target gene for miR-27a was down-regulated. SFRP1 expression is often down-regulated in breast cancer, and the up-regulation of SFRP1 expression can suppress the development of breast cancer, which validated its important role as a tumor suppressor [24]. In consistence with these findings, our study presented that SFRP1 was the target gene for miR-27a. Guo et al. [12] also identified SFRP1 as a novel target for miR-27a by dual-luciferase activity assay, and they found that miR-27a might target SFRP1 contributing to bone metabolism in hFOB cells.

To further explore the effects of miR-27a on osteosarcoma cells by targeting SFRP1, MTT assay and Transwell assay were applied to evaluate the proliferation and invasion ability of HOS and U2OS cells among seven groups. It has been reported that miR-27a plays an oncogenic role in osteosarcoma, and it stimulates the proliferation and invasion of osteosarcoma MG63 cells by targeting MAP2K4 [25]. The serum miR-27a level was elevated in osteosarcoma cells and demonstrated its associations with important clinicopathological features including advanced clinical stage of osteosarcoma, poor response to chemotherapy, as well as positive distant metastasis, indicating the oncogenic role of miR-27a in osteosarcoma [26]. Also, overexpression of miR-27a/miR-27a* contributes to the clinical metastasis of osteosarcoma by directly repressing CBFA2T2 expression [27]. Besides, the oncogenic role of miR-27a in laryngeal squamous cell carcinoma is through down-regulating PLK2, and miR-27a serves as a significant biomarker for diagnosis and therapy for this malignancy [11]. The results of our study were in agreement with the oncogenic role of miR-27a. It presented that the proliferation and invasion of HOS and U2OS cells was up-regulated in the cells transfected with miR-27a mimic. Moreover, the present study found a new target (SFRP1) for miR-27a, and the knockdown of miR-27a led to the up-regulation of SFRP1 and down-regulation of cell proliferation and invasion. These results demonstrated that miR-27a might significantly promote the proliferation and invasion of both HOS and U2OS cells by targeting SFRP1.

The article "Silencing microRNA-27a inhibits proliferation and invasion of human osteosarcoma cells through the SFRP1-dependent Wnt/β-catenin signaling pathway" was retracted in 2026. Reasons: plagiarized data; plagiarized images; overlap with other authors' work; concerns about the data.

The present study also found that miR-27a might contribute to activation of the Wnt/β-catenin signaling pathway by targeting SFRP1. The Wnt protein family can activate downstream signaling transduction pathways through combining with the receptors (Frizzled and Fz receptors) on cell surface, thus participating in the proliferation and differentiation of cells [28]. The accumulation of Wnt proteins and β-catenin protein is increased in osteosarcoma. The activation of the Wnt signaling pathway may be associated with the development of osteosarcoma due to its essential role in the differentiation of cancer stem cells [29]. SFRPs are negative modulators of Wnt signals, which plays a critical role in the pathogenesis of hematopoietic malignancies [30]. SFRP1 is located in the cysteine-rich domain (CRD) of the N-end, it might inhibit the activity of Wnt-3a thereby blocking Wnt-signaling pathway in cancer [31]. SFRP1 can combine with the Wnt receptor through the CRD region, which causes β-catenin phosphorylation and decreases its content [32]. Moreover, SFRP1 may interact with Fz receptors to form non-functional compounds [33], thereby hindering the Wnt signaling pathway and further inhibiting the proliferation and invasion of osteosarcoma cells. When SFRP1 expression was declined, the Wnt signaling pathway was activated, and signals from the Wnt could release β-catenin from its binding protein Axin to accumulate in cytoplasm and then enter into the cell nucleus. In the cell nucleus, β-catenin would combine with TCF/LEF protein, and activate the transcription and expression of target genes VEGF, cyclin D1, c-myc and matrilysin [34], thereby enhancing the proliferation and invasion ability of human osteosarcoma cells. Results of the present study revealed that the activity of TCF/LEF was elevated with the up-regulation of miR-27a, while the knockdown of miR-27a led to a decrease in the activity of TCF/LEF in osteosarcoma cells. Consequently, miR-27a might lead to the loss of SFRP1, which activates the Wnt/β-catenin signaling pathway to stimulate the proliferation and invasion of osteosarcoma cells.

In summary, the present study provided evidences for the finding that miR-27a could promote the proliferation and invasion of human osteosarcoma cells, which might be achieved by targeting SFRP1 to activate the Wnt/β-catenin signaling pathway. This finding provided a novel target for the treatment of osteosarcoma. However, the specific mechanism of miR-27a targeting SFRP1 to regulate Wnt/β-catenin signaling pathway remains to be further verified and perfected.

The article "Silencing microRNA-27a inhibits proliferation and invasion of human osteosarcoma cells through the SFRP1-dependent Wnt/β-catenin signaling pathway" was retracted in 2026. Reasons: plagiarized data; plagiarized images; overlap with other authors' work; concerns about the data.

## Abbreviations

ANOVA: analysis of variance
CRD: cysteine-rich domain
DMEM: Dulbecco’s modified Eagle’s medium
GAPDH: glyceraldehyde-3-phosphate dehydrogenase
LEF: lymphoid enhancer-binding
Luc: firefly luciferase activity
miRNA: microRNA
MTT: 3-(4,5-dimethylthiazol-2-yl)-2,5-diphenyltetrazolium bromide
PBST: phosphate buffer saline-Tween 20
PCR: polymerase chain reaction
pRL-TK: *Renilla* luciferase-thymidine kinase
Ratio of TOP-Luc/Rel: ratio of TOP-Flash Luc/*Renilla* luciferase activity
Rel value: *Renilla* luciferase activity
RT-qPCR: reverse transcription quantitative PCR
S.D.: standard deviation
SFRP1: secreted frizzled related protein 1
si-NC: negative control siRNA
TCF: T-cell factor
VEGF: vascular endothelial growth factor
3′-UTR: 3′-untranslated region
